This article has been retracted.

# Health lipid indices and physicochemical properties of dual fortified yogurt with extruded flaxseed omega fatty acids and fibers for hypercholesterolemic subjects

**DOI:** 10.1002/fsn3.1302

**Published:** 2019-12-26

**Authors:** Nazir Ahmad, Muhammad Faisal Manzoor, Umair Shabbir, Saeed Ahmed, Tariq Ismail, Farhan Saeed, MahrUn Nisa, Faqir Muhammad Anjum, Shahzad Hussain

**Affiliations:** ^1^ Institute of Home and Food Sciences Faculty of Life Sciences Government College University Faisalabad Pakistan; ^2^ School of Food Science and Engineering South China University of Technology Guangzhou China; ^3^ Institute of Food Science and Nutrition Bahauddin Zakariya University Multan Pakistan; ^4^ Department of Food and Nutrition Faculty of Life Sciences Government College University Faisalabad Pakistan; ^5^ University of The Gambia Gambia The Gambia; ^6^ College of Food and Agricultural Sciences King Saud, University Riyadh Saudi Arabia

**Keywords:** extruded powder, flaxseed, fortification, omega n‐3 fatty, yogurt

## Abstract

The aim of the present study was to prepare designer yogurt for the hypercholesterolemic subject. The yogurts were prepared from sheep and cow milk by fortifying omega fatty acids and dietary fibers of extruded flaxseed powder (EFSP). The EFSP, *Streptococcus thermophilus,* and *Lactobacillus delbrueckii sub sp bulgaricus* at 2% were added for yogurt formation. The water retention capacity, fat adsorption capacity, swelling, and solubility of EFSP were 14.38 ± 3.16 g/g, 5.31 ± 0.93 g oil/g, 25.57 ± 1.35 ml/g, and 30.53 ± 8.5%, respectively. The proximate value of protein content increased significantly from 4.12% to 5.12%. Total fat content increased from 3.50% to 4.28%. Total dietary fibers increased from 0% to 24.14%. Significant increase was observed in C18:1n9 and C18:2n6 fatty acid contents. The omega‐3 (18:3n3) was significantly increased higher as compared to other omega fatty acids in fortified yogurts. Atherogenicity index (IA: 2.23 ± 0.41 to 1.42 ± 0.23) and thrombogenicity index (IT: 1.68 ± 0.95 to 0.65 ± 0.01) were significantly decreased while the ratio of hypocholesterolemic and hypercholesteremic fatty acids (HH: 0.82 ± 0.05 to 1.29 ± 0.46) increased significantly in sheep milk yogurt. IA (2.74 ± 0.31 to 1.48 ± 0.08) and IT (1.84 ± 0.28 to 0.39 ± 0.04) were also decreased significantly while HH (0.54 ± 0.05to 1.12 ± 0.02) increased significantly in cow milk yogurt. Δ9‐desaturase (18) index was found highest (75.67 ± 8.04) in EFSP‐fortified sheep milk yogurt and lowest (62.27 ± 8.65) in cow milk yogurt while Δ9‐desaturase (16) index was maximum (6.21 ± 1.25) in cow milk yogurt and minimum (3.93 ± 1.38) in EFSP‐fortified sheep milk yogurt. Significant effect on consistency, firmness, viscosity index, and cohesiveness was also noticed in fortified yogurts. EFSP has also significant impact on colony formation of stains culture. The fortified product got good flavor and textural acceptance score. Thus; EFSP improved the health lipids quality and physicochemical characteristics. It can act as a good stabilizer and texturizer in yogurt formation and a healthy alternative for hazardous adulterants used in yogurt formation.

## Graphical abstract

EFSP improved the health lipids quality and physicochemical characteristics. It can act as good stabilizer and texturizer in yogurt formation and a healthy alternate for hazardous adulterants used in yogurt formation.

## 1 INTRODUCTION

Consumer's knowledge about functional food ingredients and their associated health benefits has been drastically increased in recent years (Brouns & Vermeer, 2000). That is why people are more conscious to have food with health benefits in their diet to increase and maintain life quality (Ahmad, Yap, Kofli, & Ghazali, 2018). In food production, the demand for functional foods with specific physiological action and health benefits of the consumer has been increased (Corbo, Albenzio, Angelis, Sevi, & Gobbetti, 2001). It is believed that dairy products have multiple health benefits due to high digestibility and nutritional value (Sadeghi, 2016). García‐Pérez et al. stated that yogurt is one of the popular dairy products that is a good food matrix and can be fortified with fruits and food ingredients (García‐Pérez et al., 2005). Since dairy products are known for their higher nutritional composition, there are lots of argument about the impact of fats on health. A plethora of scientific studies claimed that dairy products rich in fats are not suitable for human health because of the cholesterol and saturated fatty acids. It has been emphasized on the replacement of saturated fats and fortification of polyunsaturated fat in dairy products (Bermúdez‐Aguirre et al., 2011). Yogurt is one of the soft dairy products consumed by all kind of population due to its multiple health claims. The anticancer, hypocholesterolemic, diarrhea and dyspepsia treatment, detoxification of drugs, and enhancement of thiamine synthesis characteristics have been reported on yogurt consumption (Agarwal & Bhasin, 2002).

Daun et al. stated that alpha‐linolenic acid or omega‐3 fatty acids are rich in flaxseed (Daun, Barthet, Chornick, & Duguid, 2003). Generally, it consists of 50%–62% of omega‐3 fatty acids of the total fatty acids present in it and known for fiber (~10%), that is why it can be classified as a functional food (Rubilar, Gutiérrez, Verdugo, Shene, & Sineiro, 2010). So, fortification of flaxseed into dairy products like yogurt can ameliorative the texture, color, and sensorial properties. Hardness, cohesiveness, consistency, and viscosity indexes are one of the main factors to assess the textural properties of yogurt (Magenis et al., 2006).

This study was designed to fortify the sheep and cow milk with omega fatty acids and dietary fibers for yogurt formation and characterized for health lipids indices and physicochemical, textural, and sensorial properties.

## 2 MATERIAL AND METHODS

### 2.1 Procurement of materials

The milk samples of cow and sheep and stain culture of *Streptococcus thermophilus* and *Lactobacillus delbrueckii sub sp bulgaricus* and golden flaxseeds were procured from the market of Faisalabad.

### 2.2 Preparation of extruded flaxseed powder

The purpose of EFSP preparation was to improve textural and sensorial, and reduce antinutritional characteristics of final products. The twin‐screw extruder was used to extrude the flaxseed. It had a screw diameter of 36 mm with a length to diameter ratio of 24:1. It had a temperature control zone for thermal cooking with temperature measuring probe and screw speed controller. Optimization was performed using Box Behnken Design, RSM. Optimization conditions of barrel exit temperature (125°C), screw speed (125 rpm), feed flow rate (60 kg/hr), and feed moisture contents (15%) were used.

#### 2.2.1 Functional properties of EFSP

By using the methods of Femenia with some modifications, solubility, water retention capacity, swelling, and fat adsorption capacity were determined (Femenia, Lefebvre, Thebaudin, Robertson, & Bourgeois, 1997). The solubility, swelling, and water retention capacity of EFSP were measured by dispersing 2 g of EFSP for 24 hr in distilled water. Quantity of water (g) retained in the insoluble fraction of the material was used to measure the water retention capacity. Loss in the original sample on a dry weight basis (%), after the recovery of insoluble material, solubility was measured. The swelling was measured as increased bed volume after equilibration in an excess solvent. After suspending 2 g sample in sunflower oil, the fat adsorption capacity was calculated.

### 2.3 Formation of designer yogurt

Method of Walstra *et al*. with little modifications was used for yogurt preparation (Walstra, Wouters, & Geurts, 2005). Control samples were prepared by using sheep milk and cow milk. At 2% concentrations, EFSP was added to cow and sheep milk (for fortified yogurt) and then mixed uniformly (for 10 min) using a magnetic stirrer before heating. All samples were heated (85°C for 30 min) for pasteurization and cooled down to 42°C. YCX‐11 (Chr. Hansen, Denmark) starter culture (composed of *Lactobacillus delbrueckii* subsp. *bulgaricus* and *Streptococcus thermophilus*) was used. A 450 ml milk sample having a starter culture (0.2 U/L) was transferred into 500 ml Nalgene containers. Samples were kept on 42°C in an incubator for final pH of 4.6. All the samples were stored in a laboratory refrigerator at 4°C and for further analyses.

#### 2.3.1 Composition analysis

Using AACC methods, moisture content (method no; 44‐15.02), crude protein (method no; 990.03), crude fat (method no; 30‐10.01), crude fiber (method no; 962.09), and ash (method no; 942.05) were determined (AACC, 2000).

#### 2.3.2 Fatty acids profile

Fatty acid methyl esters (FAME) of samples were prepared according to the described method (Liu, 1994). Helium gas was used as a carrier, and FAME sample of 1.0 μl with gas was injected on the column at 1 ml/min rate. The column equilibrium conditions were 160°C for 0 min, and the temperature was increased to 180°C at a rate of 3°C/min with injection. The column temperature was further increased from 180°C to 220°C at 1°C/min and maintained for 7.5 min. The split ratio was 50% keeping injector and detector temperature of 240°C and 250°C, respectively. Quantitative analysis of fatty acids and composition were performed from peak area and retention time using Varian Chem Station software.

#### 2.3.3 Lipid health quality Indexes

Health lipid indexes of yogurts were assessed by calculating atherogenicity index (IA), thrombogenicity index (IT), the ratio of hypocholesterolemic and hypercholesteremic fatty acids (HH), Δ9‐desaturase (C18) index (DI (18)), Δ9‐desaturase (C16) index (DI (16)), and PUFA‐n‐6/PUFA‐n‐3 ratio. The values of these indexes indicate the quality for pro‐atherogenicity, prothrombogenicity, and risk of cardiovascular issues.

The following equations were used to calculate these indexes:

AI = (C12:0 + 4×C14:0 + C16:0)/(ΣMUFA + ΣPUFA) [23]
TI = (C14:0 + C16:0 + C18:0)/(0.5 × ΣMUFA+0.5 × ΣPUFA‐n‐6 + 3×ΣPUFA‐n‐3 + ΣPUFA‐n‐3/ΣPUFA n‐6) [24]
HH = (C18:1n‐9 + C18:2n‐6 + C20:4n‐6 + C18:3n‐3 + C20:5n‐3 + C22:5n‐3 + C22:6n‐6)/(C14:0 + C16:0)
DI (18) = 100(18:1/(18:1 + 18:0)) [25]
DI (16) = 100(16:1/(16:1 + 16:0)) [25]

PUFA‐n‐6/PUFA‐n‐3: total n‐6 PUFA fatty acids/total n‐3 PUFA fatty acids.

Σ = Summation, MUFA = monounsaturated fatty acids, and PUFA = polyunsaturated fatty acids.

#### 2.3.4 Syneresis

The proposed method of Keogh and Kennedy was used for determination of syneresis index of yogurt samples (Keogh & O'Kennedy 1998). After centrifugation (at 222 *g* for 10 min) of 20 g sample, syneresis was measured as the supernatant (whey) produced and expressed as weight %.

#### 2.3.5 Texture analysis

By using TA‐XT plus texture profile analyzer (Texture Technologies Corp), 5 kg loading cell (backward‐extrusion test), the texture of yogurt was determined. Texture analyzer parameters were modified from the template in Exponent: surface trigger force 10 g, penetration distance 30 mm, test speed 1.0 mm/s, and cylinder probe of 35 mm diameter. Analyses were performed on the yogurt samples placed in 125 ml Nalgene containers of 70 mm height and 64 mm in diameter. Consistency (N*s), firmness (*N*), viscosity index (N*s), and cohesiveness (*N*) were evaluated using the Exponent program.

#### 2.3.6 Enumeration of starter culture

*Streptococcus thermophilus* and *Lactobacillus delbrueckii subsp. Bulgaricus* enumerated according to methods of the International Dairy Foundation were used (International Dairy Federation, 1988). The *Lactobacillus delbrueckii subsp. Bulgaricus* agar (M 927) and *Streptococcus thermophilus* agar (M 948) were purchased from Lahore. All samples were mixed with peptone (0.05%) and tryptone (0.05%) in water. *S. thermophiles* were incubated in aerobic conditions at 37°C for two days on the respective agar plate. *Lactobacillus delbrueckii subsp. Bulgaricus* agar plates were incubated under a microaerobic environment at 37°C for 3 days. Colonies of *Lactobacillus delbrueckii subsp. Bulgaricus* and *Streptococcus thermophilus* were counted after incubation. Plates having colonies (30–300) were used in counting and then expressed in CFU/ml.

#### 2.3.7 Organoleptic evaluation

Yogurt samples were maintained at ambient temperature (25 ± 2°C) and presented to panelists. Five trained panelists evaluated these samples all were well familiar to yogurt. Sensory evaluation was done on the basis of 9‐point Hedonic scale.

### 2.4 Statistical analysis

All analyses were done in triplicate, and obtained results from those analyses are subjected to statistical tests by using the method of Steel, Torrie, and Dickey (1997). The difference within groups was compared using a *t* test, considering the *p*‐value <.05 as statically significant.

## 3 RESULTS

### 3.1 Compositional and Functional properties

Compositional and functional properties of EFSP are presented in Table 1. The water retention capacity, fat adsorption capacity, swelling, and solubility of EFSP were 14.38 ± 3.16 g/g, 5.31 ± 0.93 g oil/ g EFSP, 25.57 ± 1.35 ml/g, and 30.53 ± 8.5%, respectively. The nutritional composition of EFSP‐fortified designer cow and sheep milk yogurts is presented in Table 2. Total proteins ranged between 4.12% and 5.12%, total fat 3.50% and 4.28%, ash content 0.91% and 1.18%, moisture content 83.9% and 84.81%, and total dietary fibers 24.11% and 24.14% in which soluble fibers varied from 6.35% to 6.36% and insoluble fibers from 18.71% to 18.73% in plain and fortified yogurts. The significant difference was found for crude fat and total dietary fiber in yogurt samples fortified with EFSP.

**Table 1:** Functional properties of EFSP

Properties	EFSP
Water retention capacity (g/g)	14.38 ± 3.16
Fat adsorption capacity (g oil/g EFSP)	5.31 ± 0.93
Swelling (ml/g)	25.57 ± 1.35
Solubility (%)	30.53 ± 8.5

Abbreviation: EFSP, extruded flaxseed powder.

**Table 2:** Nutritional composition (%) of EFSP‐fortified designer yogurt

Indices	Sheep milk yogurt	EFSP‐fortified sheep milk yogurt	Cow milk yogurt	EFSP‐fortified cow milk yogurt
Crude fat	3.50	4.28*	3.50	4.24*
Crude proteins	4.68	5.12*	4.12	4.56
Ash	0.91	0.96	1.15	1.18
Moisture	83.9	83.99	84.7	84.81
Total dietary fibers	‐	24.11***	‐	24.14***
Soluble fiber	‐	6.36***	‐	6.35***
Insoluble fiber	‐	18.71***	‐	18.73***

Note

*On values shows a significant difference within a row.

Abbreviation: EFSP, extruded flaxseed powder.

### 3.2 Fatty acid profile of yogurts

Fatty acid profile of plain and fortified yogurts is presented in Table 3. The SFA: C10:0, C14:0, C16:0, C18:0, the MUFA: C18:1n9, and the PUFA: 18:3n3 are the predominant ones in yogurt samples tested. C16:0 was the most abundant in almost all yogurt samples and especially in EFSP‐fortified cow milk yogurt. Significant increase in fatty acids (C18:1n9 and C18:2n6) was observed in EFSP‐fortified yogurts, but highly significant improvement was noticed in 18:3n3. Sum of fatty acids and lipid health indexes are presented in Table 4. SFA (g/450 g) ranged between 11.59 ± 1.45 and 17.21 ± 2.43, MUFA 3.39 ± 0.89 and 7.78 ± 1.60, PUFA 0.58 ± 0.244 and 3.87 ± 0.92, PUFA‐n‐6 0.22 ± 0.08 and 0.88 ± 0.07, and PUFA‐n‐3 0.33 ± 0.14 and 2.99 ± 2±0.38 while the ratio of PUFA‐n‐6/PUFA‐n‐3 was 0.11 ± 0.08 to 0.85 ± 0.09 in yogurt samples.

**Table 3:** Fatty acid profile of designer yogurts (per 100 g)

Fatty acids (g)	Sheep milk yogurt	EFSP‐fortified sheep milk yogurt	Cow milk yogurt	EFSP‐fortified sheep milk yogurt
C4:0	0.13 ± 0.02	0.13 ± 0.02	0.16 ± 0.02	0.16 ± 0.02
C6:0	0.08 ± 0.009	0.08 ± 0.009	0.10 ± 0.007	0.10 ± 0.09
C8:0	0.10 ± 0.02	0.45 ± 0.02	0.047 ± 0.02	0.047 ± 0.02
C10:0	0.23 ± 0.007	0.23 ± 0.02	0.130 ± 0.004	0.131 ± 0.004
C12:0	0.12 ± 0.007	0.12 ± 0.007	0.130 ± 0.011	0.133 ± 0.011
C14:0	0.35 ± 0.009	0.35 ± 0.09	0.37 ± 0.05	0.37 ± 0.11
C14:1n5	0.01 ± 0.007	0.01 ± 0.007	0.07 ± 0.013	0.064 ± 0.004
C15:0	0.02 ± 0.02	0.02 ± 0.02	0.07 ± 0.016	0.07 ± 0.004
C16:0	0.83 ± 0.22	0.88 ± 0.12	0.96 ± 0.22	1.01 ± 0.007
C16:1n7	0.03 ± 0.01	0.036 ± 0.009	0.062 ± 0.007	0.062 ± 0.002
C17:0	0.02 ± 0.015	0.02 ± 0.02	0.04 ± 0.004	0.04 ± 0.004
C18:0	0.32 ± 0.06	0.35 ± 0.02	0.39 ± 0.16	0.42 ± 0.19
C18:1n9	0.94 ± 0.12	1.13 ± 0.27*	0.65 ± 0.22	0.84 ± 0.17*
C18:2n6	0.02 ± 0.002	0.162 ± 0.01**	0.031 ± 0.002	0.18 ± 0.024**
C18:3n6	0.004 ± 0.002	0.004 ± 0.007	0.004 ± 0.002	0.007 ± 0.002
C18:3n3	0.028 ± 0.007	0.60 ± 0.073***	0.031 ± 0.007	0.62 ± 0.19***
C20:0	0.017 ± 0.002	0.017 ± 0.002	0.009 ± 0.002	0.011 ± 0.004
C20:2	0.019 ± 0.002	0.019 ± 0.002	0.004 ± 0.002	0.004 ± 0.002
C20:3n6	0.002 ± 0.002	0.002 ± 0.002	0.016 ± 0.009	0.02 ± 0.007
C20:4n6	0.019 ± 0.004	0.019 ± 0.002	0.013 ± 0.007	0.013 ± 0.004
C20:3n3	0.011 ± 0.007	0.011 ± 0.004	0.018 ± 0.002	0.018 ± 0.002
C20:5n3	0.017 ± 0.002	0.017 ± 0.004	0.009 ± 0.002	0.009 ± 0.004
C22:0	0.017 ± 0.002	0.017 ± 0.002	0.007 ± 0.002	0.009 ± 0.002
C22:1n9	0.004 ± 0.002	0.017 ± 0.002	0.009 ± 0.002	0.011 ± 0.007
C22:2	0.02 ± 0.01	0.02 ± 0.009	0.013 ± 0.004	0.013 ± 0.004
C22:6n3	0.013 ± 0.004	0.013 ± 0.004	0.013 ± 0.007	0.015 ± 0.007
C23:0	0.011 ± 0.004	0.011 ± 0.002	0.013 ± 0.002	0.015 ± 0.004
C24:0	0.028 ± 0.007	0.028 ± 0.007	0.009 ± 0.002	0.009 ± 0.002
SFA	3.74 ± 0.32	3.82 ± 0.54	2.58 ± 0.32	2.65 ± 0.42
MUFA	1.54 ± 0.13	1.73 ± 0.35	0.75 ± 0.20	0.94 ± 0.26
PUFA	0.13 ± 0.054	0.86 ± 0.204***	0.14 ± 0.002	0.74 ± 0.21***
PUFA‐*n*−6	0.05 ± 0.018	0.20 ± 0.02***	0.062 ± 0.004	0.08 ± 0.004***
PUFA‐*n*−3	0.08 ± 0.018	0.66 ± 0.84***	0.073 ± 0.031	0.66 ± 0.013***

Abbreviations: EFSP, extruded flaxseed powder; MUFA, monounsaturated fatty acids; PUFA, polyunsaturated fatty acids; PUFA‐*n*‐3, total *n*‐3 PUFA fatty acids; PUFA‐*n*‐6, total *n*‐6 PUFA fatty acids; SFA, saturated fatty acid

**Table 4:** The ratios of fatty acids (g) and health lipid indexes of yogurts (450 g)

Indexes	Sheep milk yogurt	EFSP‐fortified sheep milk yogurt	Cow milk yogurt	EFSP‐fortified cow milk yogurt
SFA	16.85 ± 1.45	17.21 ± 2.43	11.59 ± 1.45	11.94 ± 1.90
MUFA	6.91 ± 0.60	7.78 ± 1.60	3.39 ± 0.89	4.25 ± 1.16
PUFA	0.58 ± 0.244	3.87 ± 0.92***	0.62 ± 0.01	3.31 ± 0.94***
PUFA‐*n*−6	0.22 ± 0.08	0.88 ± 0.07**	0.28 ± 0.02	0.35 ± 0.026
PUFA‐*n*−3	0.35 ± 0.08	2.99 ± 0.38***	0.33 ± 0.14	2.96 ± 0.06***
PUFA‐*n*−6/ PUFA‐*n*−3	0.619 ± 0.04	0.29 ± 0.06**	0.85 ± 0.09	0.11 ± 0.08**
AI	2.23 ± 0.41	1.42 ± 0.23**	2.74 ± 0.31	1.48 ± 0.08^**^
IT	1.68 ± 0.95	0.65 ± 0.01***	1.84 ± 0.28	0.39 ± 0.04***
HH	0.82 ± 0.05	1.29 ± 0.46**	0.54 ± 0.05	1.12 ± 0.22**
DI (18)	74.32 ± 9.92	75.67 ± 8.04	62.27 ± 8.65	66.81 ± 9.51*
DI (16)	4.03 ± 1.63	3.93 ± 1.38	6.21 ± 1.25	5.96 ± 1.39

Note

AI: atherogenic index = (C12:0 + 4×C14:0 + C16:0)/(ΣMUFA + ΣPUFA).

TI: thrombogenic index = (C14:0 + C16:0 + C18:0)/(0.5 × ΣMUFA+0.5 × ΣPUFA‐n‐6 + 3×ΣPUFA‐n‐3 + ΣPUFA‐n‐3/ΣPUFA‐n‐6).

HH: Hypocholesterolemic/hypercholesterolemic fatty acids = (C18:1 n‐9 + C18:2 n‐6 + C20:4 n‐6 + C18:3 n‐3 + C20:5 n‐3 + C22:5 n‐3 + C22:6 n‐6)/(C14:0 + C16:0).

DI (18): Δ9‐desaturase (C18) index = 100(18:1/(18:1 + 18:0)).

DI (16): Δ9‐desaturase (C16) index = 100(16:1/(16:1 + 16:0).

The superscript (^*^) on values shows significance difference within row.

Abbreviations: EFSP, extruded flaxseed powder; MUFA, monounsaturated fatty acids; PUFA, polyunsaturated fatty acids; PUFA‐n‐3, total n‐3 PUFA fatty acids; PUFA‐n‐6/PUFA‐n‐3, total n‐6 PUFA fatty acids/total n‐3 PUFA fatty acids; PUFA‐n‐6, total n‐6 PUFA fatty acids; SFA, saturated fatty acid.

### 3.3 Lipid health indexes

Lipid health indexes like AI, IT, and HH in sheep milk yogurt were observed as 2.23 ± 0.41, 1.68 ± 0.95, and 0.82 ± 0.05; in EFSP‐fortified sheep milk yogurt 1.42 ± 0.23, 0.65 ± 0.01, and 1.29 ± 0.46; in cow milk yogurt 2.74 ± 0.31, 1.84 ± 0.28, and 0.54 ± 0.05; and in EFSP‐fortified cow milk yogurt 1.48 ± 0.08, 0.39 ± 0.04, and 1.12 ± 0.022, respectively. Δ9‐desaturase (18) index was found highest (75.67 ± 8.04) in EFSP‐fortified sheep milk yogurt and lowest (62.27 ± 8.65) in cow milk yogurt while Δ9‐desaturase (16) index was maximum (6.21 ± 1.25) in cow milk yogurt and minimum (3.93 ± 1.38) in EFSP‐fortified sheep milk yogurt.

### 3.4 Syneresis and textural parameters of yogurts

The decrease in syneresis was noticed with the fortification of EFSP in both yogurts. Level of syneresis in sheep milk yogurt, EFSP‐fortified sheep milk yogurt, cow milk yogurt, and EFSP‐fortified cow milk yogurt was 27.6%, 25.7%, 28.9%, and 26.3%, respectively. All textural parameters significantly increased (*p < .*05) with the fortification of EFSP in both sheep and cow milk yogurt (Table 5). EFSP‐fortified sheep milk yogurt showed more firmness, consistency, cohesiveness, and viscosity index than EFSP‐fortified sheep milk yogurt. So, EFSP can be used as a stabilizing agent in yogurt.

**Table 5:** Textural parameters of designer yogurts

Parameters	Sheep milk yogurt	EFSP‐fortified sheep milk yogurt	Cow milk yogurt	EFSP‐fortified cow milk yogurt
Firmness (*N*)	0.86 ± 0.02	2.02 ± 0.13***	0.83 ± 0.08	1.96 ± 0.10**
Consistency (N*s)	19.92 ± 1.07	28.72 ± 2.05**	19.21 ± 1.98	25.77 ± 2.67**
Cohesiveness (*N*)	0.41 ± 0.04	2.15 ± 0.14**	0.39 ± 0.05	1.98 ± 0.08**
Viscosity index (N*s)	1.07 ± 0.09	3.25 ± 0.19**	1.04 ± 0.07	3.17 ± 0.94**

Note

*On values shows a significant difference within the row.

### 3.5 Enumeration of *S. thermophilus* and *L. delbrueckii* subsp. *bulgaricus*

The significant change in starter culture was noticed in yogurts with EFSP (Figure 1). The *S. thermophilus* count in sheep milk yogurt, EFSP‐fortified sheep milk yogurt, cow milk yogurt, and EFSP‐fortified cow milk yogurt was 2.20 × 10^8^, 2.26 × 10^8^, 2.18 × 10^8^, and 2.27 × 10^8^cfu/ml, and *L. delbrueckii subsp. Bulgaricus* count was 1.54 × 10^8^, 1.60 × 10^8^, 1.53 × 10^8^, and 1.62 × 10^8^, respectively.

**Figure 1:** shows the enumeration of S. thermophilus and L. delbrueckii subsp. bulgaricus colony formation (×108cfu/mL). EFSP: extruded flaxseed powder

### 3.6 Organoleptic evaluation

Trained panelists gave good scores to four samples. Maximum sensory scores (presented in Figure 2) were given to EFSP‐fortified sheep milk yogurt. Improvement in texture was observed by evaluators in EFSP‐fortified yogurts.

**Figure 2:** shows the score of organoleptic evaluation of yogurts performed using Hedonic 9‐point scale for sensorial parameters

## 4 DISCUSSION

Flaxseed is an emerging functional food ingredient as it has a rich source of polyunsaturated fatty acids especially α‐linolenic acid (C18:3n3) and fibers. It can possess many health benefits likewise prevention of atherosclerosis, cardiovascular disease, cancer, diabetes, osteoporosis, arthritis, and neurological and autoimmune disorders. Flaxseed oil as a functional food ingredient has been incorporated into dairy products, baked foods, muffins, juices, macaroni, meat, and pasta products (Goyal et al., 2016). EFSP‐fortified yogurts were prepared in this study. Milk samples were standardized at 3.5%, and incorporation of EFSP has ameliorated the effect of functional yogurts. Simmons et al. claimed that flaxseed has one‐third (soluble fiber) and two‐third (insoluble fiber) that are about 28 g/100 g of flaxseed. After incorporation of flaxseed powder into yogurts, total dietary fiber values were 24.11 (%) for EFSP‐fortified sheep milk yogurt and 24.14 (%) for EFSP‐fortified cow milk yogurt and these values are slightly different from Simmons et al. findings that might be due to different flaxseed species (Simmons et al., 2011).

Goh et al. stated that PUFAs such as linoleic and α‐linolenic acids are present about 80% flaxseed oil. C18:1, C18:2, and C18:3 are one of the most vital fatty acids that are necessary to maintain human health (Goh, Ye, & Dale, 2006). They found a significant difference in the content of polyunsaturated fatty acid (C18:3) between control yogurt to yogurt samples incorporated with flaxseed oil and flour. Amount of fatty acids (C18 above) was significantly higher in yogurt incorporated with flaxseed flour and oil; these observations are following the current study. SFAs and MUFAs were higher in sheep's than in cow's yogurts, although there were no significant differences in the PUFA content between plain yogurt samples and these findings are in accordance with finding of Serafeimidou, Zlatanos, Laskaridis, and Sagredos (2012).

Adding EFSP during yogurt preparation affected the textural properties of fortified yogurt. The protein content of the milk base is important for the consistency of yogurt. The higher protein content of milk contributes to a stable and consistent structure of yogurts (Guven, Yasar, Karaca, & Hayaloglu, 2005). Some other ingredients may also contribute to stabilizing yogurt gel to improve consistency. In the current study, EFSP (2%) showed more consistent values than control. So, 2% EFSP could be the optimal concentration that provides an accurate effect of viscosity building capacity of soluble components and water binding. Significant increase in firmness has been noticed in EFSP‐fortified yogurts that might be due to the higher values of total solids and the interactions of EFSP with milk protein matrix that results in more rigid and denser gel structure. Cohesiveness is also one of the important parameters to define the texture of yogurt as it assesses the quality of yogurt that a force is required to prevent the yogurt adhered to the spoon or mouth when eating the product (Costa et al., 2015). EFSP‐fortified yogurt presented higher cohesiveness values and showed a similar effect on viscosity index (Kumar & Mishra, 2004). They claimed that the addition of stabilizers at a higher rate has ameliorated effect on the growth of starter culture as the addition of EFSP also has stabilizing effect in yogurt preparation and increase in starter count was noticed in fortified yogurts.

## 5 CONCLUSIONS

The dietary guidelines regarding the milk and milk product have led to increasing the consumption of dairy products but the effect of saturated fat of dairy products imposes a serious threat to the health of the population. So, the yogurt fortified with omega and fibers from EFSP for the hypercholesterolemic population was characterized by health lipid indices and physicochemical properties. Fortification of EFSP in yogurt led to better firmness, more consistency, and better health lipid indices. It has been evaluated in this study that EFSP @ 2% can act as good stabilizer and texturizer in yogurt formation and can be a healthy alternative for hazardous adulterants used for yogurt formation. Sensorial tests also verified its good flavor and textural acceptance for consumers. After the enumeration of starter culture, the colony formation of yogurt was also improved by addition EFSP.

## CONFLICT OF INTEREST

All authors declared no conflict of interest.

## ETHICAL APPROVAL

This article does not contain any studies with human participants or animals performed by any of the authors.

## INFORMED CONSENT

For this type of study, formal consent is not required.
